RETRACTED

# The Effects of Chewing Gum on Reducing Anxiety and Stress: A Meta-Analysis of Randomized Controlled Trials

**DOI:** 10.1155/2022/8606693

**Published:** 2022-01-31

**Authors:** Jing Luo, Mengjie Xia, Chen Zhang

**Affiliations:** ^1^Taizhou Shi Zhong Yiyuan, Shanghai University of Traditional Chinese Medicine Taizhou Hospital, Taizhou 318000, Zhejiang, China; ^2^Taizhou University, Taizhou 318000, Zhejiang, China

## Abstract

There was currently no consensus on whether chewing gum should be widely instituted as a means to help reduce anxiety and stress. Chewing gum was also not included in guidelines for alleviating anxiety and stress. The purpose of this study was of two aspects: (1) to review the research progress of the relationship between gum chewing and anxiety and stress in recent years and (2) to make a meta-analysis of the effects of mastication on anxiety and stress. We conducted a meta-analysis of studies extracted from PubMed, the Cochrane Library, and Embase to identify randomized controlled trials (RCTs) evaluating the efficacy of chewing gum on anxiety, and stress was evaluated through screening, inclusion, data extraction, and quality assessment. The meta-analysis we performed was using Review Manager 5.3 software. We included a total of 8 RCTs, involving more than 400 adults over 18 years old. Compared with no chewing gum, chewing gum resulted in anxiety (MD = −0.26, 95% CI (−0.48, −0.04), *p*=0.02, *I*^2^ = 11%), where the heterogeneity was low and statistically significant. While in stress (MD = −0.27, 95% CI (−0.79, −0.25), *p*=0.31, *I*^2^ = 48%), the heterogeneity was high, and there was of no statistical significance. Based on current evidence, chewing gum is an inexpensive, well-tolerated, safe, and effective way to relieve anxiety and stress. To confirm the conclusion, we still need to conduct more randomized trials.

## 1. Introduction

The data, founded by the US National Comorbidity Survey Replication, show that the lifetime risk of any type of anxiety disorder was as high as 37.3% in females and 25.6% in males [1]. A year prevalence rate is 18.1% [2]. In recent years, the majority of Americans lived with moderate or high levels of stress, with about 44% experiencing an increase in stress in the last 5 years [3]. However, there was a close relationship between stress and anxiety. More and more evidence suggested that chronic stress may contribute to the development and progression of mental health disorders, particularly anxiety and depression [4]. Anxiety was considered to be one of the important factors that produce nonspecific responses to exposure to several stressors [5]. Chewing was thought to affect stress modification in humans; two studies suggested that the neural mechanism by which chewing gum reduces stress involves the prefrontal cortex, which then affects the hypothalamic-pituitary-adrenal axis and autonomic nervous system activity [6]. Besides, chewing was tightly linked to hedonic (emotional) systems in the brain [7]. Chewing gum was not identified as anxiety and stress management intervention in guidelines. Some clinical trials have had conflicting results on the effects of gum chewing on anxiety and stress. The results suggest that chewing gum was a cost-effective and easy to implement a way to reduce stress and get more done [8]. Chewing gum also has been associated with reduced anxiety [9], and a recent report proved that long-term chewing gum was effective in reducing stress, anxiety, depression, and improving test scores in school nursing students [10]. Conversely, some studies showed chewing gum cannot reduce acute stress or anxiety [11, 12]. Experiments by Smith, Gray, and Sketchley-Kaye et al. demonstrated that cortisol increased after chewing gum [8, 9, 13]. After searching relevant literature, we found two factors which causes the change of cortisol: (1) chewing force affects the salivary cortisol level, a stress marker of the hypothalamic-pituitary-adrenal axis. (2) strong chewing force is more effective than weak chewing force in increasing cortisol [2, 13, 14]. Scholey et al. suggested that chewing time was also a factor in cortisol [15]. We think chewing gum modulates cortisol levels, which in turn reduces anxiety and stress due to changes in cortisol levels. Due to intervention intensity was only found in Scholey's study, we could not conduct a subgroup analysis. Both Allen and Smith suggested that interventions longer than two weeks reduced stress more than interventions lasting for one day [16, 17].

RETRACTED

In view of the growing literature on the use of gum chewing interventions to reduce anxiety and stress in adults, we conducted this meta-analysis to synthesize the available evidence. Our objective was to examine the relationship between gum chewing and anxiety and stress.

## 2. Methods

For meta-analysis reporting, we referred to the Preferred Reporting Items for Systematic Review and Meta-Analyses (PRISMA) recommendations [18]. The meta-analysis was registered on PROSPERO: CRD42021243550.

What is worth our attention is the relationship between chewing gum, cortisol, anxiety, and stress. Stress has been identified as a psychological factor that leads to elevated cortisol levels [4]. At the same time, cortisol has been considered a biological marker of stress and anxiety [19]. Cortisol dysregulation has been associated with anxiety [20]. We found the hypothalamic-pituitary-adrenal (HPA) axis was activated in acutely stressful situation. Activation of the HPA axis triggers the hypothalamus to release corticotropin releasing hormone (CRH) which in turn leads to the release of adrenocorticotropin hormone (ACTH) from the pituitary and finally glucocorticoids, including cortisol, from the adrenals [21]. Therefore, cortisol has gone up.

### 2.1. Search Strategy

Literature searchers were performed using PubMed, Cochrane Library, and EMBASE with the key terms “chewing gum, anxiety, stress” until the end of March 2021. There were no restrictions on language or geographical location. The detail search strategy is given in Table 1.

### 2.2. Selection Criteria

In the meta-analysis, trials were included that met the following criteria: (1) participants: adult patients (>18 years); (2) intervention group: use of chewing gum; (3) control group: no chewing gum; (4) outcome measures: report at least one of the relevant outcome data mentioned in Table 2; (5) study design: randomized controlled trial (RCT). We excluded observational, quasirandomized, crossover, or cluster-randomized trial designs and trials that did not report any outcomes of interest to this review.

### 2.3. Data Extraction

Two investigators (JL and CZ) independently reviewed the full manuscripts of eligible studies and extracted information into an electronic database, including the age and sex of the subjects, country, the type of gum, the assessment scale, and intervention time. We extracted the results of the following experimental results: anxiety and stress. Disagreements were resolved by discussion with a third reviewer (MJ X). Missing or not found data from studies deemed eligible were sought from the authors via e-mail request.

### 2.4. Assessment of Methodological Quality

Two reviewers independently evaluated RCTs quality and risk of bias following the quality checklist supplied in the Cochrane Handbook for Systematic Reviews of Interventions [22]. The authors examined six domains: method of randomization, allocation concealment, blinding, completeness of outcome data, selective reporting of outcomes, and other bias. The risk of bias in each domain was categorized as low, high, or unclear. Unclear indicated a piece of insufficient information to evaluate the risk of bias. The discrepancy was resolved by consensus, as shown in Figure 1.

### 2.5. Statistical Analysis

The articles selected for quantitative analysis were performed using Review Manager 5.3 software from the Cochrane Collaboration. For binary data variables, the odds ratio (OR) with a 95% confidence interval (CI) was calculated, and the summated outcomes of the continuous variables were expressed as a standardized mean difference (SMD). Heterogeneity was evaluated using the chi-square test, with significance set at *p* < 0.05, and quantified [23] using *I*^2^. In case of significant heterogeneity, only the results of the random-effects model were reported. Since the number of the literature was less than ten, we did not conduct a heterogeneity test. The reviews of the authors' judgments were categorized as low-risk, high-risk, or unclear-risk of bias. A forest plot was created to summarize the meta-analysis study results. Due to the limited literature included, a bias analysis of funnel plots was not performed.

RETRACTED

## 3. Results

Figure 2 shows the flowchart for the search of articles. Eight randomized controlled trials evaluating a total of 494 adults over 18 years old allocated to either a chewing gum group or a control group. The effects of gum chewing on anxiety were mentioned in five articles and stress in seven. The characteristics of the included trials are given in Table 2. These studies were published between 2009 and 2019. Five studies were conducted in the UK, two are in Austria, and one in Turkey. For gum chewing, the chewing gum group was given spearmint-flavored, sugar-free gum [9, 11, 20], one was given extra spearmint and gum base [16], one was given sugarless [10], or sugar-free gum [23], and unclear [19].

### 3.1. Anxiety

In anxiety, 8 studies reported gum chewing, involving 394 adults. The overall effect was calculated with the random-effects model owing to high heterogeneity. The combined results showed that (SMD = −0.27, 95% CI (−0.49, −0.04), *p*=0.02, *I*^2^ = 12%). Chewing gum is effective for reducing anxiety, as shown in Figure 3.

### 3.2. Anxiety Subgroup Analysis

For the intervention time, the random-effects model was used to calculate the total effects, and the comprehensive results showed that lasted more than 1 day (SMD = −0.31, 95% CI (−0.66, 0.03), *p*=0.15, *I*^2^ = 24%) and lasted less than 1 day (SMD = −0.25, 95% CI (−0.58, 0.09), *p*=0.08, *I*^2^ = 24%). Both were with low heterogeneity. There was no significant difference and correlation in the length of intervention. This may have something to do with the fact that the intervention time of several articles was less than 30 minutes (9, 11, 26), as shown in Figure 4.

For the anxiety scale, considering the different evaluation forms used, the random-effects model was adopted to calculate the total effects, and the comprehensive results showed State-Trait Anxiety Inventory (STAI) (SMD = −0.46, 95% CI (−0.89, −0.04), *p*=0.03, *I*^2^ = 0%), Hospital Anxiety and Depression Scale (HADS) (SMD = −0.05, 95% CI (−0.33, 0.23), *p*=0.70, *I*^2^ = 1%), and Depression Anxiety Stress Scale (DASS) (SMD = −0.49, 95% CI (−0.91, −0.06), *p*=0.02, *I*^2^ = 0%). Three anxiety scales were used in the 5 studies, and the overall heterogeneity was low. Using the HADS scale, the experimental group was ineffective, as shown in Figure 5.

RETRACTED

For the sample size, the random-effects model was used to calculate the total effects, and the comprehensive results showed that for sample size <50 (SMD = −0.46, 95% CI (−0.89, −0.04), *p*=0.03, *I*^2^ = 0%) and sample size >50 (SMD = −0.20, 95% CI (−0.48, 0.08), *p*=0.15, *I*^2^ = 23%). The overall heterogeneity is low. A sample size <50 is considered valid, as shown in Figure 6.

### 3.3. Stress

In stress, 10 studies reported gum chewing, involving 458 adults. The overall effect was calculated with the random-effects model owing to high heterogeneity. The combined results showed that (SMD = −0.30, 95% CI (−0.49, −0.12), *p*=0.001, *I*^2^ = 0%) chewing gum is effective on stress, as shown in Figure 7.

### 3.4. Stress Subgroup Analysis

For the intervention time, the random-effects model was used to calculate the total effects, and the comprehensive results showed that lasted more than 1 day (SMD = −0.23, 95% CI (−0.51, 0.05), *p*=0.10, *I*^2^ = 0%) and lasted less than 1 day (SMD = −0.23, 95% CI (−0.47, 0.02), *p*=0.07, *I*^2^ = 0%). Both had no heterogeneity. There was no significant difference and correlation in the length of intervention, as shown in Figure 8.

For the sample size, the random-effects model was used to calculate the total effects, and the comprehensive results showed that when sample size <50 (SMD = −0.27, 95% CI (−0.59, −0.06), *p*=0.11, *I*^2^ = 15%), there was low heterogeneity. When sample size >50 (SMD = −0.32, 95% CI (−0.56, −0.09), *p*=0.0007, *I*^2^ = 0%), there was no heterogeneity. A sample size more than 50 is considered valid, as shown in Figure 9.

## 4. Discussion

Before this, no meta-analysis has been found on the correlation between gum chewing and anxiety and stress, and we are not sure to what extent the research has been carried out on this subject. This meta-analysis found that chewing gum might be beneficial for improving anxiety and stress when compared to untreated controls. Also, our subgroup analysis was divided into groups according to the duration of intervention, anxiety scale, and sample size. We found the duration of the intervention was considered to be ineffective for anxiety and stress, and the size of the sample had different effects. In addition, the use of the HADS test proved no advantage to the experimental group over the control group, while the use of the STAI and DASS test showed that the experimental group had advantages over the control group.

RETRACTED

We performed a subgroup analysis with the mastication intervention time of a day as the boundary, and the results showed that the claim of chewing time on the effect of anxiety and stress was not valid. The alleviating heterogeneity of gum chewing on anxiety was *I*^2^ = 12%, and the alleviating heterogeneity of gum chewing on stress was *I*^2^ = 0%. The low heterogeneity was attributed to the small age gap among the healthy participants, the same intervention methods, and the similar sample size. For the anxiety scale, stress scales were used, and the heterogeneity was *I*^2^ = 12%. The low heterogeneity may be due to the fact that all three forms are authoritative measures of anxiety. STAI was one of the most widely studied and used measures of general anxiety [24]. HADS and DASS provide good indicators of depression and anxiety, often with regular screening for psychological distress [25]. In addition, the related law of large numbers holds that the central limit theorem was valid as random samples become large enough, usually defined as *n* = 30 [26]. The sample sizes of these experiments were all greater than 30, and we performed a subgroup analysis of the sample size of the experiment, which yielded inconsistent results in the anxiety sample size less than 50 which is valid. In the pressure, the sample size more than 50 is valid. The reason for this difference was that in the subgroup analysis of anxiety, the sample size of the two groups was significantly different. The sample size less than 50 was 58, and the sample size more than 50 was 166.

The advantages of our review include a comprehensive search of qualified studies, application systems and clear eligibility criteria, careful consideration of study quality, and rigorous analytical methods. On the other hand, the authors were well aware of some of the limitations of this review. First, the quality of the included trials was not necessarily high due to randomization techniques, allocation concealment, and blinding, which are all potential sources of bias. Second, anxiety and stress were studied separately and the different evaluation scales used in the literature. Third, the personal habits of men and women were different and need group research. Because previous research had shown that women are more likely to chew gum than men [27]. In these 8 articles, only men were included in Walker's study [28], and unfortunately, we are unable to subgroup men and women based on the available data. Fourth, different recruitment methods, inclusion criteria, and data collection techniques might also lead to differences in outcome indicators. Last, the taste of gum and the relaxing effects of chewing the sweet and flavored gum (the SAP of the sapodilla tree) were first suggested by Hollingworth in 1939 [29]. It was known that menthol may have a soothing effect on anxiety and stress [30, 31], similar to what Hollingworth has mentioned.

RETRACTED

When planning further studies, particular attention should be paid relating to the following points: (1) using recommended, comparable, reliable, and valid measures of anxiety and stress outcomes; (2) age and gender should be taken into consideration when selecting the survey population; (3) ensure concealment of allocation and blinding of outcome assessors to interventions; and (4) the taste and intensity of chewing gum were also worth considering.

## 5. Conclusion

More and more people were experiencing anxiety and psychological stress from all aspects caused by cultural changes, socioeconomic changes, and stress from work and study. Current meta-analyses suggested that chewing gum was an inexpensive, safe, well-tolerated, and widely available anxiety and stress reliever, although the mechanism of action is unclear.

In addition, the results of subgroup analysis supported that intervention time and evaluation scale had little influence on the heterogeneity of experimental results. Due to the low methodological quality of the studies, it was not conclusive. Future researchers should consider more detailed questions when studying the effects of gum chewing on anxiety and stress. We need to ensure concealment of allocation and blinding of outcome assessors to interventions and consider the taste and intensity of chewing gum [32].

## Figures and Tables

**Figure 1:** Risk of bias summary.

**Figure 2:** The flowchart for the search of articles.

**Figure 3:** Anxiety forest plot.

**Figure 4:** Anxiety timing forest plot.

**Figure 5:** Anxiety scale forest plot.

**Figure 6:** Anxiety sample forest plot.

**Figure 7:** Stress forest plot.

**Figure 8:** Stress timing forest plot.

**Figure 9:** Stress sample forest plot.

**Table 1:** Search strategy.

Chewing gum and anxiety, PubMed search strategy
#1 “Chewing Gum” [MeSH terms]
#2 “Gum Chewing” [title/abstract] OR “Gum^*∗*^” [title/abstract]OR “chewing” [title/abstract]
#3 #1 OR #2
#4 “Anxiety” [MeSH terms]
#5 “Anxiety disorder” [title/abstract] OR “Anxie^*∗*^”[ title/abstract] OR “Anxious^*∗*^”[ title/abstract] OR “Obsess^*∗*^”[title/abstract] OR “Stress” [title/abstract] OR “Distress”[title/abstract] OR “Stress disorder” [title/abstract]
#6 #4 OR #5
#7 #3 AND #6

**Table 2:** Summary of study characteristics.

	Country	Sample (*N*)	Mean age	Male (%)	Intervention			Scale	Outcome	
					Treatment group	Intervention time	Evaluation time		Anxiety	Stress
Allen, 2015	UK	126	29 ± 6.7	0.31	Chewing gum	1 day	1 day	HADS, self-report questionnaires	No affect	Cannot reduce
Gray, 2012	UK	40	20.25	50	Chewing gum	>1 week	1 day	HADS		Nonsignificant
Scholey, 2009	Australia	40	21.98 ± 4.79	20	Chewing gum	20 min	1 day	VAMS, STAI	Reduce	Reduce
Sketchley-Kay, 2011	UK	36	20.4	13.9	Chewing gum	25 min	1 day	VAMS,STAI	Reduce	
Smith, 2012	UK	72	19.5	8.33	Chewing gum	2 weeks	2 weeks	HADS, PSS	Nonsignificant	Reduce
Torney, 2009	UK	40	20.9	50	Chewing gum	5 min	5 min	VAMS		Cannot reduce
Walker, 2015	Austria	40	25.2 ± 4.3	100	Chewing gum	17 min	17 min	VAMS,SIMKAP		Cannot reduce
Yaman-Sözbir, 2019	Turkey	100	20.5 ± 0.9	13.9	Chewing gum	7 days, 19 days	7 days, 19 days	DASS	Reduce	Reduce

RETRACTED

## Data Availability

The data used to support the findings of this study are included within the article.
